# Dynamic Prediction of Internet Financial Market Based on Deep Learning

**DOI:** 10.1155/2022/1465394

**Published:** 2022-09-21

**Authors:** Zixuan Zhang, Xiaojun Jia, Shan Chen, Menggang Li, Fang Wang

**Affiliations:** ^1^Business School, The University of Hong Kong, Pok Fu Lam, Hong Kong; ^2^National Academy of Economic Security, Beijing Jiaotong University, Beijing 100044, China; ^3^Beijing Center for Industrial Security and Development Research, Beijing Jiaotong University, Beijing 100044, China; ^4^Beijing Laboratory of National Economic Security Early-warning Engineering, Beijing Jiaotong University, Beijing 100044, China

## Abstract

P2P lending is an important part of Internet finance, which is popular among users because of its efficiency, low cost, wide range, and ease of operation. The problem of predicting loan defaults is affected by many factors, such as the linear and nonlinear nature of the data itself and time dependence and multiple external factors, which have not been well captured in the previous work. In this paper, we propose a multiattention mechanism to capture the different effects of various time slices and various external factors on the results, introduce ARIMA and LSTM to capture the linear and nonlinear characteristics of the lending data respectively, and establish a Time Series Multiattention Prediction Model (MAT-ALSTM) based on LSTM and ARIMA. This paper uses the Lending Club dataset from the United States to prove that our model is superior to ANN, SVM, LSTM, GRU, and ARIMA models in the prediction effect of MAE, RMSE, and DA.

## 1. Introduction

Internet finance [1] refers to a new financial business model in which traditional financial institutions and Internet companies use Internet technology information and communication technology to achieve financing, payment, investment, and information intermediary services. Compared with traditional finance, Internet finance has the advantages of high efficiency, low cost, wide scope, and convenient operation, but it is also accompanied by higher risks. At present, e-banking, online banking, and mobile banking are widely promoted by commercial banks, all belonging to the category of Internet [2] finance. However, the model of Internet finance has, to a certain extent, caused problems such as low threshold in the financial market, enhanced market liquidity, and difficulties in supervision.

In 2017, China has surpassed the United States to become the largest online lending transaction time in the world. The comprehensive transaction volume of online lending platforms reached 1163.98 billion yuan. According to the World Bank's forecast, the global crowdfunding market will reach $300 billion in 2025. Behind the rapid development of Internet finance, it bears many risks [3], such as high credit risk, high network security risk, policy stay, and lack of supervision, which has led to chaos in the industry and unscrupulous elements engaging in illegal fund raising and fraud. Since 2020, P2P online lending platforms such as “Taojindi,” “Youyi.com,” and “Antai Zhuoyue” have been exposed to “runaway” incidents.

As a basic part of the P2P market, P2P online lending platforms accept social loan requests and provide people with investment opportunities. Compared to traditional bank loans, P2P loan origination relies heavily on the borrower's credit as collateral, and P2P loans are funded by thousands of active lenders on the platform. These characteristics mean that P2P loans are unsecured, and the potential for property loss is high.

Therefore, tracking and predicting the lending market dynamics of Internet finance can predict and grasp the system risk of the platform promptly, and developing appropriate default risk management methods is significant to the system, platform, and users. However, the dynamic tracking and prediction of lending data is difficult due to the high liquidity, uncertainty, and volatility of the lending market. In addition, the number of influential variables in the online environment has increased, and the relationships of various time series have become more complex [4].

The prediction of P2P lending data is a typical multifactor time series prediction problem [5]. This problem differs from traditional forecasting problems in many ways. Specifically, it is manifested in the following points. (1) The data have obvious time sequence and strong time correlation with linear and nonlinear characteristics. (2) Historical data of different periods have different influences on the data to be predicted, manifesting a greater influence between series with closer time and a smaller influence between series with farther time. (3) Various factors have different effects on time series data. For example, if a lender has a higher annual income and a higher credit rating, the loan may be smaller and the default rate on the loan is lower. However, the impact is different, so the prediction process also needs to consider the impact of different factors on the results.

Most traditional time series forecasting algorithms model financial P2P lending data as time variable series. Among them, the ARIMA model is a classic time series forecasting method, which can better reflect the linear characteristics of time series data. However, time series data in finance in general consists of two components: linear and nonlinear [6]. A single ARIMA model can hardly handle the nonlinear variation of financial lending data completely and effectively, and it needs to be combined with other algorithms. In the deep learning algorithm, due to its special network structure, the LSTM model is faster and easier to converge to the optimal solution than the traditional neural network when dealing with time series problems. It is very suitable for processing time series data such as financial loan data.

Based on the above analysis of the P2P data prediction problem, this paper proposes a new MAT-ALSTM (Time Series Multiattention Prediction Model Based on LSTM and ARIMA) model, which can be effectively applied in multifactor finance time series forecasting, and the contributions of this paper can be summarized as follows:

1. Modeling loan data as multifactor time series data, fully considering the time correlation of P2P loan markets, and the linear and nonlinear dependencies between time series data model the linear and nonlinear properties of the lending data with ARIMA and LSTM, respectively.
2. This paper proposes a multiattention mechanism to integrate input variables, where according to the different influences of historical data in different periods on the prediction period, a time series attention mechanism is proposed. Aiming at the different influences of varying time sequence features of input variables on the target value, a sequence feature attention mechanism is proposed.
3. Given the characteristics of P2P loan market data, this paper uses long and short-term memory neural networks to capture the time correlation of loan data and proposes a time series P2P market loan default prediction model MAT-ALSTM based on a multiattention mechanism.
4. This paper conducts a large number of experiments on a real dataset, which proves the superiority of the MAT-LSTM model proposed in this paper in terms of RMSE, MAE, and DA compared with LSTM, GRU, and other models.

The rest of this paper is described as follows. In Section 2, we review the traditional time series forecasting methods and the application of deep learning to time series problems. In Section 3, we introduce the problem of loan data time series prediction, long short-term memory neural network, and attention mechanism. In Section 4, we propose a time series financial market dynamic prediction model MAT-ALSTM based on a multiattention mechanism and introduce the internal structure of the model in detail. In Section 5, we conduct prediction experiments and analyze the results.  Section 6 summarizes the work of this paper.

## 2. Literature Review

In this section, we review the previous work on modeling and prediction of financial lending data in terms of (1) traditional machine learning-based prediction work and (2) deep learning network-based prediction work.

Some research works are based on traditional statistical methods and machine learning. Traditional statistical models analyze and predict default risk by finding the optimal linear combination of input variables, mainly including logistic regression, discriminant analysis, risk index models, and probabilistic models. For example, Serrano-Cinca and Gutiérrez-Nieto [7] demonstrated the advantages of multivariate discriminant analysis and logistic regression over neural networks in medium-term bankruptcy prediction of “Tunisian” firms. Chen et al. [8] used the partial least squares discriminant analysis (PLS-DA) model to predict the US banking crisis and obtained results close to SVM. Malekipirbazari and Aksakalli [9] used the borrower data of the P2P lending platform “Paipaidai,” used the information gain technology to filter the features, and constructed a logistic regression model to evaluate the borrower's credit risk. Ma [10] proposed a random forest-based classification method to predict the status of borrowers, which outperformed the FICO credit score. Niu et al. [11] used the LightGBM algorithm to predict the default rate, which performed better than the XGBoost algorithm and also found that the most important factor affecting the borrower's repayment was the loan details.

There are different kinds of deep learning models: deep multilayer perceptron, RNN, LSTM, CNN, restricted Boltzmann machines, and autoencoder [12]. Deep learning analyzes historical data of online lending and explores the inner logic behind the data, which in turn enables the assessment and prediction of credit risk. For example, Wang and Ni [13] proposed a deep dense convolutional network for social lending repayment prediction. Many works are based on LSTM and other models for financial time series forecasting. For example, Chen et al. [14] used the long short-term memory (LSTM) model for the first time to analyze P2P. For sequence data, this model has greater potential than traditional time series models. Cao et al [15] used the LSTM model to improve the accuracy of stock return forecasts by 12.9%. Molina et al [16] showed better performance in stock market price prediction by combining the LSTM model and empirical mode decomposition. In the field of e-commerce, LSTM models can effectively predict the future behavior of customers [17]. Yan et al. [18] improved the genetic algorithm by using the long short-term memory network LSTM and constructed the fitness function in a new way. The algorithm can effectively avoid the local optimal trap of the genetic algorithm and has better global search performance, and it promotes the combination of intelligent scheduling with intelligent manufacturing and e-commerce. Compared with BP neural network, traditional RNN, and RNN-improved LSTM deep neural network, LSTM can effectively predict stock market time series and have higher prediction accuracy [19]. In addition, the attention mechanism improves the generalization ability of the network and improves the average prediction accuracy of systemic risk indicators in China's financial market [20]. Meanwhile, hybrid models are used in some papers. Yuan et al. [21] combined CNN and LSTM, CNN is used to make the quantitative stock selection strategy for judging stock trends, and then LSTM is used to make the quantitative timing strategy for improving the profits. Batres-Estrada [22] proposed a novel depth and breadth neural network, which is a combination of RNN and CNN. Hochreiter and Schmidhuber [23] combined DBN and MLP to construct a stock portfolio by predicting the monthly log returns of each stock and selecting only those stocks that are expected to perform better than the median. In addition, new methods have been used in some studies.

From the analysis of existing work, we can draw the following conclusions:

1. Traditional statistical methods and machine learning methods only consider several features of a single lending data without considering the temporal coupling relationship existing in the data itself. Besides, many machine learning methods cannot capture the nonlinear relationships among time series data well, resulting in poor model coupling.
2. Some time series deep learning models can handle time series data better; however, many models do not consider the interactions between adjacent one-step or multistep time slices and fail to capture the time dependence well.
3. Few works consider the importance of different sequence features on the prediction results. Machine learning and deep learning models are able to handle multifeature data; however, different features have different impacts on lending default rates, yet many models fail to capture them well.

Based on the above analysis, this paper proposes a time series prediction model based on a multiattention mechanism, using ARIMA and LSTM algorithms to deal with both linear and nonlinear features of financial loan data to fully consider the time series and the different importance of sequence features to the results.

## 3. Method

### 3.1. Financial Lending Time Series Forecasting Problem

A time series is a sequence of observations recorded in chronological order over a fixed time interval. The prediction problem is to fit a model to predict the future values of the series, taking into account the past values. Let *X*={*X*_1_, *X*_2_,…, *X*_*T*_,} be the historical data of a time series, *H* be the desired prediction range, and the task is to predict the next value of the series {*X*_*T*+1_, *X*_*T*+2_,…, *X*_*T*+*H*_,}. $\hat{X}=\left\{\hat{X_{1}},\hat{X_{2}},\ldots ,\hat{X_{T}}\right\}$ is the vector of predicted values, and the goal is to minimize the prediction error.

Time series forecasting refers to using historical data in the past period to predict data in the future, including continuous forecasting (numerical forecasting and range estimation) and discrete forecasting (event forecasting and data classification). The financial lending time series forecasting problem can be summarized as follows.

Given a period *τ*, each financial time series includes *F* eigenvalues, and then, all the financial time series features in the *τ* The financial period can be shown as *X*^*τ*^=(*X*_1_^*τ*^, *X*_2_^*τ*^,…, *X*_*N*_^*τ*^) ∈ *R*^*N*×*F*^, where *X*_*i*_^*τ*^ ∈ *R* represents all eigenvalues of the *i*-th time series, *N* is the total number of time series, and we set *y*_*i*_^*τ*^ ∈ *R* to represent the characteristics of financial variables in the future *τ* time period. The financial prediction model can be expressed, using the past financial time series features *X*^*τ*^ to predict the financial variable features *y*_*i*_^*τ*^ ∈ *R* in the future *τ* time period.

### 3.2. LSTM

LSTM (long short-term memory) [24] is an improved RNN (recurrent neural network) model. The basic unit of the LSTM model is a memory block, which includes a memory cell and three control memories. The gate structure of the cell state include the forget gate, the input gate, and the output gate. The forget gate decides to forget the useless historical information from the memory unit state, the input gate decides the influence of the current input data on the memory unit state, and the output gate decides the output information, thus selectively forgetting the unimportant information and reinforcing the important information of the previous sequence.

The structure of the LSTM memory module is shown in Figure 1. Suppose *x*_*t*_ represents the input vector at time *t*, *h*_*t*−1_ represents the output at time *t*-1, *W*_*f*_, *W*_*i*_,*W*_*C*_, *W*_*o*_, *U*_*f*_, *U*_*i*_, *U*_*C*_, *U*_*o*_ and *W*_*f*_, *W*_*i*_, *W*_*C*_, *W*_*o*_, respectively, represent the weight matrix and the bias vector, and the process of the memory module for state update and information output is as follows.

First, the forget gate forgets useless historical information:

(1) $$\begin{array}{c} f_{t}=\sigma \left(W_{f}x_{t}+U_{f}h_{t-1}+b_{f}\right)\text{.} \end{array}$$

Then, the input gate performs state updates based on the input data and historical information:

(2) $$\begin{array}{c} i_{t}=\sigma \left(W_{i}x_{t}+U_{i}h_{t-1}+b_{i}\right)\text{,} \end{array}$$

(3) $$\begin{array}{c} {\tilde{C}}_{t}=\tanh\;\left(W_{C}x_{t}+U_{C}h_{t-1}+b_{C}\right)\text{,} \end{array}$$

(4) $$\begin{array}{c} C_{t}=f_{t}*C_{t-1}+i_{t}*{\tilde{C}}_{t}\text{.} \end{array}$$

Finally, the output gate outputs the information at the current moment:

(5) $$\begin{array}{c} o_{t}=\sigma \left(W_{o}x_{t}+U_{o}h_{t-1}+b_{o}\right)\text{,} \end{array}$$

(6) $$\begin{array}{c} h_{t}=o_{t}*\;\tanh\;\left(C_{t}\right)\text{,} \end{array}$$

where *σ* is the logistic sigmoid function, and *f*_*t*_, *i*_*t*_, and *o*_*t*_, respectively, represent the output state of the forget gate, the input gate, and the output gate at time *t*, and *C*_*t*_ represents the state of the memory cell at time *t*.

### 3.3. Attention Mechanism

The attention mechanism in deep learning [25] is a resource allocation scheme that allocates computational resources to more important tasks while solving the information overload problem when computational power is limited. In neural network learning, the more parameters a model has, the more expressive the model is, and more information is stored in the model, but this will bring about the problem of information overload. Then, by introducing an attention mechanism, focusing on the information that is more critical to the current task among the input data, reducing the attention to other information, or even filtering out irrelevant information, the information overload problem can be solved and the efficiency and accuracy of task processing can be improved.

The attention mechanism in the time series problem divides the learning model into two parts. First, the encoder composed of a single-layer or multilayer RNN encodes the input sequence according to the time relationship, which is used to learn the predependency and postdependency relationship and the current state representation of the known sequence, and generates the state representation of the current time. During the process of cyclic encoding, we get the state of the last moment and keep it, and this state retains the dynamic information of the input sequence and the current sequence state, which is denoted as vector *C*. Secondly, a decoder is composed of neural network units of similar structure, which converts the encoding vector *E* into time series information with a prediction length of *τ*. (*y*_1_, *y*_2_, *y*_3_,…, *y*_*j*−1_) is a vector obtained by common mapping, and the output value at time *j* is the predicted value at the corresponding time, namely,

(7) $$\begin{array}{c} E=F\left(x_{1},x_{2},x_{3},\ldots ,x_{\tau }\right)\text{,} \end{array}$$

(8) $$\begin{array}{c} y_{i}=G\left(E,y_{1},y_{2},y_{3},\ldots ,y_{j-1}\right)\text{.} \end{array}$$

In the traditional model, the context vector *E* used at each moment of decoding is fixed. This structure does not incorporate the principle of different information at different times into the model [19]. Therefore, this paper designs the attention mechanism and combines the structure of the encoder and decoder, and a method of sequential attention mechanism is proposed. For each prediction time *j*, the encoder obtains a dynamic context vector *E*_*j*_ with different attention information so that the decoding process can pay more attention to the prediction content of the current time and important historical information specifically by

(9) $$\begin{array}{c} E_{j}=F\left(x_{1},x_{2},x_{3},\ldots ,x_{\tau },h,h_{j-1}^{\prime }\right)\text{,} \end{array}$$

(10) $$\begin{array}{c} y_{i}=G\left(E_{j},y_{1},y_{2},y_{3},\ldots ,y_{j-1}\right)\text{,} \end{array}$$

where *F* represents the process of combining the attention mechanism with the encoder part, *h*_*j*−1_′ is the hidden state of the previous step at time *j* of the decoder, and *h* is the hidden state set of the encoder.

## 4. MAT-ALSTM

In this section, on the basis of III, a multiattention mechanism-based time series financial market dynamic prediction model MAT-ALSTM is proposed. The model structure is shown in Figure 2:

The MAT-LSTM model consists of the following modules, including a data preprocessing module, a time series modeling module, and a prediction module. Among them, the data preprocessing module processes the raw financial loan time series data for missing values and outliers and normalizes the data to meet the needs of model training. The time series modeling module consists of two parts: ARIMA modeling and LSTM modeling. Among them, ARIMA modeling mainly extracts the linear part in the loan time series data, and LSTM modeling mainly extracts the nonlinear part in the loan time series data. In the LSTM module, we also introduce a multiattention mechanism to distinguish the different effects of different time series and sequence features on the results. Finally, the prediction module mainly combines the modeling results of ARIMA and the modeling results of LSTM to obtain the final prediction results.

### 4.1. Data Preprocessing

This work uses lending data disclosed by the US P2P lending platform Lending Club as the data source. The data range is from June 2008 to December 2015. A total of 2,260,701 data are available in the raw data. The data preprocessing process mainly deals with the data in the original data. For missing values and outliers, first, outlier detection is performed on the data, outliers are regarded as missing values, and the missing values are filled by using Lagrangian interpolation. Secondly, we calculate the average default rate of new loans per month as the dependent variable, and the formula is as follows:

(11) $$\begin{array}{c} Default\;rate\;of\;monthly\;new\;loan=\frac{Defaults\;of\;monthly\;new\;loans}{Total\;monthly\;new\;loans}\text{.} \end{array}$$

In order to make the data more suitable for the model training process, we standardized the data by max-min on columns. The normalization process is as follows:

(12) $$\begin{array}{c} X_{norm}=\frac{X-X_{\min}}{X_{\max}-X_{\min}}\text{.} \end{array}$$

Financial loan data have both linear and nonlinear features. Denote the loan data as *D*_*t*_, which can be decomposed into a linear part *l*_*t*_ and a nonlinear part *n*_*t*_, which are recorded as

(13) $$\begin{array}{c} D_{t}=l_{t}+n_{t}\text{.} \end{array}$$

In the preprocessing process, the data are first processed for missing values. For the original dataset of 144 columns of features, there are 60 columns of features containing missing values and 43 columns of features with a percentage of true values above 30%, so we first remove the features with missing values above 30%. The digitized features are filled using the mean or median of other samples, and the nondigitized features are predicted using Sklearn. For outliers, we take the approach of using the mean rather than the outlier samples.

### 4.2. ARIMA Modeling

The ARIMA model [26] is a differential autoregressive moving average model, which includes two processes: AR autoregression (*p*) and MA moving average regression (*q*). The general form of this model is given as

(14) $$\begin{array}{c} y_{t}=\mu +\overset{p}{\underset{i=1}{\sum }}\gamma_{i}y_{t-i}+\epsilon_{t}+\overset{q}{\underset{i=1}{\sum }}\theta_{i}\epsilon_{t-i}\text{,} \end{array}$$

where *p* is the lag order of the autoregressive process, *q* is the lag order of the moving average process, *μ* is the constant term coefficient, and *ϵ*_*t*_ is the random disturbance term sequence, which is shown as the white noise sequence *ϵ*_*t*_ ~ *WriteNoise*(0, *σ*_*t*_^2^). The ARIMA model requires that the event sequence must be a stationary sequence during modeling. For nonstationary time series data, the d-order difference should be performed before modeling. Therefore, the complete difference autoregressive moving average process *ARIMA*(*p*, *d*, *q*) is introduced in the introduction. The model after the lag factor is given as

(15) $$\begin{array}{c} \left(1-\overset{p}{\underset{i=1}{\sum }}\varphi_{i}L^{i}\right){\left(1-L\right)}^{d}y_{t}=c+\left(1+\overset{q}{\underset{i=1}{\sum }}\theta_{i}L^{i}\right)\varepsilon_{t}\text{,} \end{array}$$

where *L* represents the lag factor, which is defined as *L*^*n*^*y*_*t*_=*y*_*t*−*n*_, and (1 − *L*)^*d*^ is the d-order difference operation.

### 4.3. Time Series Modeling

First, we use the ARIMA model to model the data, then fit the training data, and make predictions, and the output prediction result is recorded as *X*_*t*_′, and the residual error can be obtained as

(16) $$\begin{array}{c} R_{t}=D_{t}-X_{t}^{\prime }\text{.} \end{array}$$

In view of the different influences of historical data of different time periods on the prediction period and the different influences of different sequence features of input variables on the target value, we propose a multiattention mechanism.

The hidden state at different times has different degrees of attention. In the time dimension, an attention mechanism based on the historical state of the lending market is constructed as follows:

(17) $$\begin{array}{c} e_{tj}=V_{a}^{T}\tanh\;\left(W_{a}h_{j-1}^{\prime }+U_{a}h_{t}\right)\text{,} \end{array}$$

(18) $$\begin{array}{c} e_{tj}^{\prime }=softmax\left(e_{tj}\right)\text{,} \end{array}$$

where *h*_*j*−1_′ is the hidden state of the model training in the previous stage; *h*_*t*_ is the loan market state at time *t* in the model training; *V*_*a*_^*T*^, *W*_*a*_, and *U*_*a*_ are all learnable parameter matrices. *e*_*tj*_ represents the degree of influence of the state of the loan market at time *t* in the encoder on the output of the state at the current predicted time *j*. Finally, the softmax function is used to normalize *e*_*tj*_ to obtain the weight factor of the current prediction of the state of the loan market at each historical time. *e*_*tj*_′ is the attention value in the time dimension.

Different sequence features have different degrees of attention. In the sequence feature dimension, an attention mechanism based on the time series features of the lending market is constructed as follows:

(19) $$\begin{array}{c} p_{tj}=V_{p}^{T}\tanh\;\left(h_{j-1}^{\prime }W_{p}\right)+b_{p}\text{,} \end{array}$$

(20) $$\begin{array}{c} p_{tj}^{\prime }=softmax\left(p_{tj}\right)\text{,} \end{array}$$

where *h*_*j*−1_′ is the hidden state of the model training in the previous stage; *V*_*p*_^*T*^, *W*_*p*_, and *b*_*p*_ are all learnable parameter matrices; *p*_*tj*_ represents the sequence feature of the lending market at time *t* in the encoder for the influence degree of the state output of *j* at the current prediction time; and finally, normalize *p*_*tj*_ through the softmax function so as to obtain the weight factor *p*_*tj*_′ of different sequence features to the current prediction, that is, the attention value in the sequence feature dimension.

The nonlinear components in the loan data are hidden in the residual sequence *R*_*t*_. Next, the LSTM model is used to train and predict the residual sequence, and the predicted value *E*_*t*_′ of the residual sequence is obtained.

### 4.4. Prediction Result

After preprocessing, the model will be trained by the ARIMA model, and the training result *X*_*t*_′ will be used as the output of the linear feature capture module, followed by using the original loop data *D*_*t*_ to do residual processing with *X*_*t*_′, which is noted as *R*_*t*_ which is the nonlinear part of the borrowing data, followed by adding a temporal attention mechanism to the temporal dimension of the data and a multifactor attention mechanism to the feature dimension, followed by using LSTM for the capture of that part of the features. Finally, the results are linearly summed to obtain the final prediction results.

Combining the linear prediction value *X*_*t*_′ of the ARIMA time series model and the nonlinear prediction value *E*_*t*_′ of the LSTM model, the final prediction value *Result*_*t*_′ is

(21) $$\begin{array}{c} {Result}_{t}^{\prime }=X_{t}^{\prime }+E_{t}^{\prime }\text{.} \end{array}$$

## 5. Experiment

### 5.1. Lending Club Dataset

In the experiment, the desensitized data published on the official website of Lending Club were selected for the experiment. The time range is from 2008 to 2015. The data include personal information, loan information, and credit information. The loan status variable is the main focus of this paper. It has seven states: fully paid, charge off, default, current, in grace period, late (16–30 days), and late (31–120 days). In this paper, we argue that all statuses should be considered as default except for the status of full payment.

As shown in Figure 3, we count the borrowings and defaults in the raw data from January 2009 to December 2009.

### 5.2. Model Evaluation

Models built on time series data must make accurate forecasts in two dimensions of metrics: prediction accuracy and prediction trend accuracy. Therefore, we choose root mean square error (RMSE), mean absolute error (MAE), and orientation accuracy (DA) as the evaluation metrics in this paper. Among them, RMSE and MAE are used to evaluate the prediction accuracy of model predictions, and DA is used for evaluating the forecast trend accuracy of models' predictions. Formulas of the three statistical indices are as follows:

(22) $$\begin{array}{c} RMSE=\sqrt{MSE}=\sqrt{\frac{1}{m}\overset{m}{\underset{i=1}{\sum }}{\left(y_{i}-\hat{y_{i}}\right)}^{2},} \end{array}$$

(23) $$\begin{array}{c} MAE=\frac{1}{m}\overset{m}{\underset{i=1}{\sum }}\left|\left(y_{i}-\hat{y_{i}}\right)\right|\text{,} \end{array}$$

(24) $$\begin{array}{c} DA=\frac{1}{m}\overset{m}{\underset{i=1}{\sum }}a_{i},a_{i}=\left\{\begin{array}{cc} 1\text{,} & \left(y_{i+1}-y_{i}\right)\left({\hat{y}}_{i+1}-y_{i}\right)>0\\ 0\text{,} & \left(y_{i+1}-y_{i}\right)\left({\hat{y}}_{i+1}-y_{i}\right)\leq 0\text{,} \end{array}\right. \end{array}$$

where $\hat{y_{i}}$ is the prediction result of the model, *y*_*i*_ is the true value of the origin sample data, and *m* is the number of samples.

### 5.3. Experimental Set-Up

In the following, we explain the experimental set-up for the models involved in this paper, as shown in Tables 1 and 2.

### 5.4. Results and Analysis

We use ARIMA [26], SVM [27], ANN [28], LSTM [24], and GRU [29] models for comparison, and Table 3 shows the performance of this model on the loan default rate from January 2014 to December 2015, and the optimal result has been bolded.  Figure 4shows the numerical prediction of the loan default rate of each model from January 2014 to December 2015.

Here, we will briefly introduce the baseline model. ARIMA [26] is an autoregressive integrated moving average model, which analyzes and forecasts time series data with perfection and accuracy. SVM [27] is a class of generalized linear classifier that performs binary classification of data in a supervised learning manner. ANN [28] simulates the neuronal activity with a mathematical model and is an information processing system based on mimicking the structure and function of neural networks in the brain. LSTM [24] and GRU [29] are variants of recurrent neural networks, which can better capture the nonlinear temporal data properties.

From Table 3, we know that the indices of MAT-ALSTM model on the three metrics are 0.049, 0.043, and 0.7, respectively, which achieved optimal results compared to ARIMA and GRU models and achieved a good enhancement effect, as shown in Table 4.

In order to compare the prediction accuracy of each model more conveniently, we draw the following model comparison chart, as shown in Figure 5. It can be observed from the image that the MAT-ALSTM model curve obtains the lowest value in the RMSE and MAE indicator and the maximum value in the DA metrics.

Next, we show the prediction results of the six models at some time points with the real data, as shown in Figure 4, and it can be observed approximately that the prediction results of the MAT-ALSTM model are closer to the real situation compared to the other models.

As shown in Table 1 and Figures 4 and 5, the results of this paper are analyzed as follows.

1. The MAT-MLSTM model proposed in this paper has better prediction effect than the LSTM and GRU models
2. The SVM model and ANN model do not take into account the time series characteristics of loan data, so the prediction effect is poor
3. Compared with the ARIMA model and LSTM model, the MAT-ALSTM model has significantly better prediction results because the MAT-ALSTM model captures the linear and nonlinear characteristics of the loan data, respectively
4. Although the LSTM model and GRU model consider the time series characteristics of loan data, they do not consider the important difference between time series and series characteristics, while the MAT-ALSTM model fully considers the above characteristics and introduces many attention mechanisms, so the prediction effect is better

## 6. Conclusion

P2P lending is one of the important components of Internet finance. Accurate lending data prediction is of great significance for applications such as platform construction, user evaluation, and system upgrades. This paper takes the loan default rate of users as the research object, fully considers the linear and nonlinear characteristics of the loan data, and proposes a multiattention model MAT-ALSTM based on LSTM and ARIMA, which can handle the time series in loan data well and fully capture the importance of different time series and sequence features to the prediction results. The experimental results show that the MAT-ALSTM model in this paper has a better prediction effect than GRU, LSTM, and other models.

Theoretically, our model provides a new perspective for processing and prediction of time series data, i.e., starting from the linear and nonlinear characteristics of time series data itself and using the corresponding mechanisms to capture and merge the results to complete the prediction.

In practice, our model has better prediction results compared with LSTM and GRU models, and the model complexity is not too high, and it can be used as a base model to compose components of deeper models, which are more accurate compared with simple RNN and its variants.

In the future, we will try to combine the model with other domains, such as transportation and retail to verify its usability in other domains. Besides, in this paper, we use a self-attentive mechanism to describe the importance of different time slices and features, and we will also try the attention mechanism design approach. Finally, the interpretability problem of the model has been a bottleneck that hinders the application of deep learning, so we will try to improve the interpretability of the model.

## Figures and Tables

**Figure 1:** Structure diagram of LSTM memory module. *f*_*t*_: the forget gate, *i*_*t*_: the input gate, *o*_*t*_: the output gate, *C*_*t*_: the state of the memory cell at time *t*, *h*_*t*−1_: the output at time *t* − 1.

**Figure 2:** MAT-ALSTM model architecture.

**Figure 3:** Total borrowings and defaults from January 2009 to December 2009.

**Figure 4:** Predictions of loan default rates from January 2014 to December 2015. (a) The prediction result from January 2014 to December 2014. (b) The prediction result from January 2015 to December 2015.

**Figure 5:** Comparison of prediction accuracy of each model.

**Table 1:** Experimental set-up of LSTM and GRU models.

Hyperparameters	LSTM	GRU
Hidden layers	5	5
Optimization algorithm	Adam	Adam
Learning rate	0.001	0.001
Epoch	Early stopping	Early stopping
Mini-batch	15	15
Dropout rate	0.005	0.005

**Table 2:** Experimental setup of ARIMA, SVM, and ANN models.

Parameters	ARIMA	Hyperparameters	SVM	Hyperparameters	ANN
AR	1	Kernel	Linear	Nodes	32
Difference	0	Gamma	0.001	Learning rate	0.001
MA	1	Cost	25	Optimizers	Adam
—	—	—	—	Activation	Relu

**Table 3:** Comparison between MAT-ALSTM and the baseline model.

Evaluation	RMSE	MAE	DA
ARIMA	0.113	0.104	0.455
SVM	0.104	0.09	0.547
ANN	0.073	0.059	0.636
LSTM	0.055	0.05	0.636
GRU	0.055	0.047	0.7
MAT-ALSTM	**0.049**	**0.043**	**0.7**

**Table 4:** Performance improvement of MAT-ALSTM compared to other models.

	RMSE (%)	MAE	DA (%)
Compare with ARIMA	130.6	141.85	53.8
Compare with SVM	112.2	109.3%	27.9
Compare with ANN	48.9	37.2%	10
Compare with LSTM	12.2	16.2%	10
Compare with GRU	12.2	9.3%	0

## Data Availability

All data used in our study could be accessed by the request to the corresponding author.
